The article "Mechanistic Research into the Effects of the Jianpi Xiaozhi Formula on Liver Injury in Diabetic Rats" was published in 2022. Journal: Evid Based Complement Alternat Med.

# Mechanistic Research into the Effects of the Jianpi Xiaozhi Formula on Liver Injury in Diabetic Rats

**DOI:** 10.1155/2022/7490747

**Published:** 2022-07-20

**Authors:** Zhang Yuanyuan, Liu Huaizhen

**Affiliations:** Department of Endocrinology, Geriatrics Center, The First Affiliated Hospital of Anhui University of Traditional Chinese Medicine, 117 Meishan Road, Hefei 230009, Anhui, China

## Abstract

**Objective:**

The purpose of this study was to explore the mechanism of Jianpi Xiaozhi Formula (JPXZF) action in attenuating liver injury in a rat model of type 2 diabetes mellitus (T2DM).

**Methods:**

A rat model of T2DM was established. Forty-eight male Sprague–Dawley (SD) rats were randomly allocated to six groups: healthy untreated rats (normal control (NC)), rats with diabetes mellitus (DM), diabetic rats treated with low-dosage JPXZF (DM + JL), diabetic rats treated with an intermediate JPXZF dosage (DM + JM), diabetic rats treated with high-dosage JPXZF (DM + JH), and diabetic rats treated with 4-phenylbutyric acid (PBA) (DM + PBA). The rats in each group were given the indicated drugs for 8 weeks, and pathological changes in the liver tissues of each rat group were observed by haematoxylin-eosin (HE) staining. Reverse-transcription polymerase chain reaction (RT-PCR) and Western blotting (WB) were performed to determine the expression of glucose-regulated protein 78 (GRP78), activating transcription factor 6 (ATF6), family with sequence similarity 134, member B (FAM134B), P62, Beclin-1, and light chain 3II/I (LC3II/I) genes and proteins in the liver tissues of the rats in each group. Immunofluorescence was used to observe changes in FAM134B expression.

**Results:**

After successfully establishing the rat model, RT-PCR assays revealed that, compared with those in the NC group rats, the expression levels of GRP78, ATF6, and P62 mRNA in the livers of the DM group rats were significantly increased, and the relative expression levels of FAM134B and Beclin-1 mRNA were significantly decreased. Compared with that in the DM group, the relative expression of GRP78, ATF6, and P62 mRNA in the liver of the rats in each JPXZF intervention group was decreased in a dosage-dependent manner, and the relative expression of FAM134B and Beclin-1 mRNA was increased significantly (*p* < 0.05). WB indicated that, compared with that in the NC group rats, the LC3II/I protein expression ratio in the liver of the DM group rats was significantly reduced, and the LC3II/I protein expression ratio in the liver of the rats in each JPXZF intervention group was significantly increased. In addition, the expression of the other measured proteins was consistent with that of the corresponding mRNA measured by RT-PCR (*p* < 0.05). The immunofluorescence assay results showed that FAM134B changes were consistent with the results obtained by RT-PCR and WB (*p* < 0.05).

The article "Mechanistic Research into the Effects of the Jianpi Xiaozhi Formula on Liver Injury in Diabetic Rats" was published in 2022. Journal: Evid Based Complement Alternat Med.

**Conclusion:**

Jianpi Xiaozhi Formula may be effective in treating liver injury in diabetic rats by regulating autophagy induced by endoplasmic reticulum stress (ERS).

## 1. Introduction

Type 2 diabetes mellitus (T2DM) is a chronic metabolic disease characterized by disordered sugar, fat, and protein metabolism caused by insufficient islet secretion of insulin or insulin resistance (IR). Recent statistics have shown that the global incidence of T2DM was 425 million in 2017, and this number is expected to increase to 629 million by 2045 [1]. Specifically, the incidence of diabetes mellitus (DM) in China is 10.9%, which is the highest in the world [2]. The onset of T2DM is affected by many chronic diseases, such as obesity, hypertriglyceridaemia, and nonalcoholic fatty liver. Among these causes, the relationship between nonalcoholic fatty liver disease (NAFLD) and T2DM has been of particularly high concern in recent years. NAFLD is characterized by an abnormal accumulation of liver cell fats and IR. NAFLD worsens over time, pathologically progressing from simple steatosis to nonalcoholic steatohepatitis (NASH), then to liver fibrosis followed by cirrhosis, and finally hepatocellular carcinoma [3]. The incidence of NAFLD in T2DM patients is as high as 70% [4]. A large sample analysis of 473,374 people showed that compared with that for patients with neither form of diabetes, the risk of death associated with NAFLD in T2DM patients increased from two to threefold and was highest for those with cardiovascular disease or liver disease [5]. Reflecting on these data, at the American Diabetes Annual Meeting, a new statement suggested that “DM is a liver disease.”

Complications in the pathogenesis of T2DM in patients with NAFLD are unknown. Generally, IR has been considered the initial cause of liver steatosis with inflammatory factors and oxidative stress thought to be secondary factors in liver cell injury that leads to persistent endoplasmic reticulum stress (ERS). Moreover, the interaction of various factors has been suggested to lead to lipid peroxidation, which aggravates liver steatosis and leads to NAFLD [6]. ERS has been recently confirmed to be involved in the occurrence and development of T2DM and NAFLD by contributing to lipid metabolism disorder, IR and oxidative stress [7, 8]. When the ER is hyperstressed, insoluble or toxic protein aggregates are formed in the ER cavity, and the function and structure of ER calcium pumps can be damaged, which triggers the autophagy pathway to clear the retained protein aggregates and other molecules damaging the ER [9]. Autophagic clearance of damaged or redundant cell contents relies on the lysosome pathway. A specific type of autophagy, ER-autophagy, changes ER function and structure. Specifically, the ER undergoes fragmentation, and these ER fragments are engulfed by the forming autophagosomal membrane, which removes them from cells. Therefore, moderate levels of ER-autophagy can prevent the occurrence and development of diseases; however, hyperactivated ER-autophagy can clear normal ER or trigger cellular reactions through signalling pathways that aggravate pathological changes in the body. Spanish scholar González-Rodrguez et al. [10] found that in ERS the expression levels of stress-related markers glucose-regulated protein 78 (GRP78) and activating transcription factor 6 (ATF6) were significantly increased in 49 NAFLD patients, as determined by pathological biopsy samples. In particular, the expression level of the autophagy-related molecule Beclin-1 was significantly decreased, and the level of light chain 3II/I (LC3II/I) was significantly increased. These results suggested that autophagic flux was damaged in NAFLD patient livers and that restoring autophagic flux may slow NAFLD progression.

The article "Mechanistic Research into the Effects of the Jianpi Xiaozhi Formula on Liver Injury in Diabetic Rats" was published in 2022. Journal: Evid Based Complement Alternat Med.

Family with sequence similarity 134, member B (FAM134B) is an activated receptor in ER-autophagy. FAM134B includes an LC3-binding domain, which can bind to the autophagy-related protein LC3. After LC3 is recruited, FAM134B promotes ER-autophagy [11]. Liang et al. [12] pointed out that FAM134B reshapes ER morphology, regulates autophagy clearance and ER turnover, and maintains intracellular homeostasis. Liao et al. [13] proved that Z36 is a previously undiscovered small-molecule inhibitor of the Bcl2-2 protein family expression that upregulates the expression levels of FAM134B and LC3. Overexpression of FAM134B can induce ER-autophagy and upregulate LC3 expression levels. Yuan et al. [14] found that FAM134B was highly expressed in obese pigs. Cai et al. [15] pointed out that overexpression of FAM134B promoted adipocyte autophagy and reduced the number of mitochondria, thus affecting obesity. Later, the weight and white adipose tissue mass in mice with specific FAM134B overexpression were increased significantly, and these mice simultaneously developed hyperglycaemia and severe IR. Obesity, DM, and NAFLD are chronic metabolic diseases; therefore, we hypothesized that ERS is associated with the occurrence and development of T2DM with NAFLD as a comorbidity by inhibiting autophagy and that the ER-autophagy receptor FAM134B plays an important role in this process.

T2DM with NAFLD is not universally defined in ancient literature. In general, “Xiaoke” in traditional Chinese medicine describes diabetes, and NAFLD is the category of “accumulation.” Considering the clinical data and literature review results, we believe that “stagnation of liver depression, spleen deficiency, and phlegm block” is the common etiological bases of T2DM with NAFLD; therefore, according to traditional Chinese medical practice, Jianpi Shugang and Huatan Quyu are prescribed. Jianpi Xiaozhi Formula (JPXZF), a compound prepared by Chief Physician Liu Huaizhen in our hospital, shows the combined effects of Jianpi Shugang and Huatan Quyu. JPXZF was originally used to reduce glucose and lipid levels in patients with T2DM with dyslipidaemia [16, 17]. To discover the mechanism underlying the effect of this compound in enhancing glucose and lipid metabolism, our research group established a dyslipidaemia rat model of T2DM. The compound was shown to increase SOD activity; reduce the MDA content, which reduced oxidative stress [18]; and reduce the expression of inflammatory factors (chemerin, TNF-*α* [19], MCP-1, NF-KB [20]), played an anti-inflammatory role. After long-term clinical application, JPXZP was found [21, 22] to reduce blood sugar and lipids in patients with T2DM with NAFLD through its anti-inflammatory and antioxidative stress effects. Another study revealed that JPXZF attenuated atherosclerosis [23] and reduced intima-media thickness [24] in patients with T2DM and macroangiopathy by downregulating MMP-9 and IL-1*β* expression levels.

The article "Mechanistic Research into the Effects of the Jianpi Xiaozhi Formula on Liver Injury in Diabetic Rats" was published in 2022. Journal: Evid Based Complement Alternat Med.

A diet consisting of high sugar and high fat is often a key pathological factor in NAFLD. In this study, a high-sugar and high-fat feed combined with an intraperitoneal injection of low-dose streptozotocin (STZ) were used to induce a T2DM rat model. This model required a short modelling time, a high success rate, relatively slight direct damage to the liver, a relatively long rat survival time, and a stable course; therefore, it was suitable for the study of diabetic liver injury [25]. The effect of JPXZF on the expression of ER-autophagy markers in the model rat liver tissue was measured, and the specific mechanism of action was investigated to provide a greater scientific basis for its application in clinical treatment.

## 2. Materials and Methods

### 2.1. Materials

JPXZF was provided by the First Affiliated Hospital of Anhui University of Traditional Chinese Medicine. The granules were crushed for later use. The components were radix pseudostellariae, 15 g; jiang banxia, 9 g; dried tangerine peel, 6 g; poria cocos, 10 g; bamboo shavings, 10 g; safflower, 5 g; wolfberry fruit, 10 g; fried white peony root, 10 g; raw atractylodes rhizome, 10 g; and earthworm, 6 g. As determined by high-performance liquid chromatography (HPLC) analysis, the JPXZF sample consisted of polysaccharides, guanosine, atractylenolide I, and atractylenolide III at 7.6% [26], 0.02%, 0.014%, and 0.027%, respectively [27]. 4-PBA was purchased from the Macklin Company (Shanghai, China). STZ was purchased from Sigma (St. Louis, USA). Pentobarbital was purchased from Beijing Dingguo Changsheng Biotechnology Co. Ltd. (Beijing, China). High-sugar and high-fat feed (10% sucrose, 10% lard, 1% cholesterol, 0.3% sodium cholate, and 78.7% basic feed) was provided by the Qingyuan Experimental Animal Center of Anhui Province.

The article "Mechanistic Research into the Effects of the Jianpi Xiaozhi Formula on Liver Injury in Diabetic Rats" was published in 2022. Journal: Evid Based Complement Alternat Med.

### 2.2. Animals

Forty-eight healthy male Sprague–Dawley (SD) rats (8 weeks old with an average weight of 180 ± 20 g) were provided by the Qingyuan Experimental Animal Center of Anhui Province. All the rats had continuous access to food and water in their cages. The feeding environment was always well ventilated with an indoor temperature of 18–25°C and relative humidity of 40–70%. The experiment was approved by the Experimental Animal Ethics Committee of Anhui University of Traditional Chinese Medicine.

### 2.3. Experimental Planning

Forty-eight healthy male SD rats were randomly allocated to a normal control (NC) group (*n* = 8) and a DM group (*n* = 40) after one week of adaptive feeding with a basic diet. The rats in the NC group were fed basic feed for 8 weeks. The other 40 rats were used to establish a rat model of T2DM according to a method described in the literature [28]. Specifically, the rats were first fed a high-sugar and high-fat diet for 8 weeks and then fasted for 12 hours. Then, they were intraperitoneally injected with 30 mg/kg STZ; the NC group was intraperitoneally injected with the same dosage of citric acid buffer. Three days after the injection of STZ, blood was removed from the tail vein of the DM group rats and the blood sugar was measured at least twice and was ≥16.7 mmol/L, which confirmed the successful establishment of the T2DM rat model [29]. Forty T2DM model rats were randomly allocated to a new DM group (*n* = 8), a group that was treated with low-dosage JPXZF (DM + JL, *n* = 8), a group treated with an intermediate-dosage JPXZF (DM + JM, *n* = 8), a group treated with high-dosage JPXZF (DM + JH, *n* = 8), and a group treated with PBA (DM + PBA, *n* = 8). Rats in the NC and DM groups were administered normal saline by gavage following the procedure outlined in Pharmacological Experimental Methodology, which was edited by Professor Xu Shuyun [30]. The JPXZF dosage administered to the rats was 6.3-fold greater than that prescribed to human adults, as calculated on the basis of the equivalent surface area ratio of the experimental animals to that of a 60-kg human adult. For example, a 9 g/kg/d JPXZP dosage was given to rats in the intermediate-dose group. The JPXZF dosage for rats in the high-dosage group was 18 g/kg/d, which is twofold the high dosage given to human adults in the clinic. The 4.5 g/kg/d JPXZF dosage given to rats in the low-dosage group was 0.5-fold that of the low-dosage given to adults in the clinic. As the positive control, 2.5 mg/kg/d PBA was administered to rats by gavage [31]. All the drugs were administered orally for 8 weeks.

The article "Mechanistic Research into the Effects of the Jianpi Xiaozhi Formula on Liver Injury in Diabetic Rats" was published in 2022. Journal: Evid Based Complement Alternat Med.

### 2.4. Measurement of Serum Indexes and Drug Retention in Tissue Samples

After 8 weeks of JPXZF intervention, all the rats fasted for 12 hours with water freely accessible. Then, the mouse body weight was measured, and the mice were anaesthetized with pentobarbital (45 mg/kg) administered intraperitoneally before 4-5 ml of abdominal aortic blood was removed. Each blood sample was poured into an Eppendorf (EP) tube, which was centrifuged for 10 min at 3000 rpm to separate the serum and plasma. The serum fasting blood glucose (FBG), triglyceride (TG), total cholesterol (TC), alanine aminotransferase (ALT), and aspartic acid aminotransferase (AST) levels were measured with a Hitachi 7600A-020 automatic biochemical analyser. Fasting insulin (FINS) levels were detected by radioimmunoassay. After the rats were killed, the abdominal cavity was opened, the liver was removed, and washed repeatedly with normal saline. Then, a portion of the right-lobe liver tissue was fixed in 10% formalin, and the pathological changes in the liver tissue were observed after haematoxylin-eosin (HE) staining. Another small piece of the liver tissue was placed in a tin paper box with the embedding agent OCT and stored in a −80°C freezer before immunofluorescence detection. The remaining liver tissue was immediately diced and placed into two sterile cryopreservation tubes, immediately frozen in liquid nitrogen, and then quickly transferred to a −80°C freezer for use reverse-transcription-polymerase chain reaction (RT-PCR) and Western blotting (WB).

### 2.5. Haemoxylin-Eosin (HE) Analysis

The rat liver tissue was fixed in 10% formalin for 24 hours, embedded in paraffin, and cut into sections with a thickness of 3 *µ*m. The sections were treated with HE from a staining kit (Solarbio, Beijing, China) according to the manufacturer's instructions. The histological changes in liver tissues were assessed under a light microscope (Olympus, Tokyo, Japan).

### 2.6. Immunofluorescence Detection

The rat liver tissue was fixed in 4% paraformaldehyde for 30 min, washed three times with a phosphate buffer solution, sealed with goat serum (Zsbio, Beijing, China) for 1 hour, and incubated overnight in a wet box with an anti-FAM134B antibody (Abcam, Cambridge, England) at 4°C, rewarmed in a wet box at 37°C for 30 min, and treated with fluorescein II at 37°C (Shanghai, China) incubated in the dark for 1 hour, stained with DAPI (Beyotime, Shanghai, China) for 5 min, sealed with an anti-fluorescence quenching sealing solution (Beyotime, Shanghai, China), and photographed with a fluorescence microscope (Motic, Shenzhen, China). Using Image-Pro Plus Version 6.0 (IPP) image analysis software, the integrated optical density (IOD) of each slice was calculated, and the IOD value was used to express the quantification index.

The article "Mechanistic Research into the Effects of the Jianpi Xiaozhi Formula on Liver Injury in Diabetic Rats" was published in 2022. Journal: Evid Based Complement Alternat Med.

### 2.7. Reverse-Transcription Polymerase Chain Reaction (RT-PCR)

Total RNA in the rat liver tissue was extracted by TRIzol (Invitrogen, Carlsbad, CA). The RNA concentration was determined, and 1 *µ*g of RNA was added to reverse transcriptase (TaKaRa, Dalian, China) to transcribe the mRNA into cDNA, which was stored at −80°C. Then, a Novo Start SYBR Super Mix Plus (Novo Protein, Jiangsu, China) kit was used for real-time fluorescence quantification and amplification PCR. For RT-PCR, the samples were incubated in 96-well optical plates at 95°C for 1 min, followed by 40 cycles at 95°C for 20 s and 60°C for 1 min. The threshold cycle (Ct) method was used to calculate the mRNA expression (2-ΔΔCT). The following primer sequences, designed by Sangon Biotech (Shanghai, China), were used: GRP78 (F: 5′-ATGTCAGAAAGGACAACAGAGC-3′, R: 5′-TTTCATGGTAGAGCGGAACA-3′); ATF6 (F: 5′-GCAGGTGTATTACGCTTCGC-3′, R: 5′-TCTTCGGTCTTGTGGTCTTGT-3′); p62 (F: 5′-CGAAAGCTGACGCTGTTCAT-3′, R: 5′-GGAGGACGGTACAAATCCATTA-3′); FAM134B (F: 5′-AGGCTTACTTGTCAGGTGGC-3′, R: 5′-CAGAAACGTCAGGTTTTGCTT-3′); and *β*-actin, the internal control (F: 5′-CCCATCTATGAGGGTTACGC-3′, R: 5′-TTTAATGTCACGCACGATTTC-3′).

### 2.8. Western Blotting (WB)

RIPA cell lysis buffer (Beyotime, Shanghai, China) was used to lyse the liver tissue cells, and then, total protein was extracted and the protein concentration was determined. After sodium dodecyl sulfate-polyacrylamide gel electrophoresis (SDS-PAGE), the proteins were transferred to a PVDF membrane (Millipore, Bedford, MA). The PVDF membrane was removed from the transfer apparatus and placed into 5% skim milk, which blocked it, for 1-2 hours. Then, the membrane was incubated with primary antibodies (Abcam, Cambridge, England) overnight, followed by incubation with secondary antibodies (Zsbio, Beijing, China). Finally, an enhanced chemiluminescence (ECL) hypersensitive luminescence kit (Thermo, Shanghai, China) was used to detect the proteins.

The article "Mechanistic Research into the Effects of the Jianpi Xiaozhi Formula on Liver Injury in Diabetic Rats" was published in 2022. Journal: Evid Based Complement Alternat Med.

### 2.9. Statistical Analysis

The SPSS 21.0 statistical software was used for data analyses. Kolmogorov–Smirnov tests were performed to determine the normality of all the data. The data following a normal distribution are presented by $\bar{x}\pm S$. The groups were compared by single-factor variance analysis. *P* < 0.05 indicates a statistically significant difference.

## 3. Results

### 3.1. Histopathological Analysis

In the NC group, the rat hepatic lobule structure was clear and complete; that is, the hepatic cords were neatly organized, the liver cells were arranged radially around the central vein, the size was uniform, the nuclei were round, and the cell shape was regular. Moreover, no fatty degeneration of the liver cells or inflammatory cell infiltration in the portal area was observed. The sinus hepaticus was clearly visible. However, in the DM group, the structure of the hepatic lobule was destroyed, the hepatic cords were disordered, and the liver cells exhibited an irregular morphology and swelling indicative of diffuse bullous steatosis and ballooning. Finally, lipid deposits were evident in the liver cells, and inflammatory cells had infiltrated the portal area and lobule. In summary, the rats in the DM group presented with liver injury. Compared with the DM group, all the JPXZF intervention groups (DM + JL, DM + JM, and DM + JH groups) presented with a reduced degree of fatty liver-related changes in liver cells, including fewer intracellular lipid droplets and lower inflammatory cell infiltration. Notably, the differences were the most profound between the high-dosage intervention and DM groups (Figure 1).

### 3.2. Comparison of General Serological Indexes of the Rats in Different Groups

Compared with those in the NC group, the levels of serum FBG, FINS, TG, and TC and the body weight of the rats in the DM group were significantly increased, and compared with those in the DM group, the levels of serum FBG, FINS, TG, and TC and the body weight in each JPXZF intervention group were markedly decreased with increasing drug dosage, and the levels of serum FBG, FINS, TG, and TC and the body weight in the DM + PBA group were also decreased significantly. Compared with those in the DM + JL group, the levels of serum FBG, FINS, TG, and TC and the body weight in the DM + JH group were further decreased (*p* < 0.05). Compared with those in the NC group, no significant difference in ALT or AST levels was found in the DM group, JPXZP intervention groups, or DM + PBA group, which indicated that the early intervention of drugs did not cause hepatotoxicity and was safe (Table 1).

### 3.3. Effect of JPXZF on Endoplasmic Reticulum Stress (ERS)

The results of an RT-PCR showed that compared with those in the NC group rats, the relative expression levels of GRP78 mRNA and ATF6 mRNA in the liver of the DM group rats were significantly increased, and the relative expression levels of GRP78 mRNA and ATF6 mRNA in the liver of the JPXZF intervention group rats decreased, in a dosage-dependent manner, compared with those in the DM group rats but were higher than those of the NC group rats. Compared with those in the DM + JL group rats, the relative expression levels of GRP78 mRNA and ATF6 mRNA in the liver of the DM + JH group rats were further decreased (*p* < 0.05) (Figure 2(a)). The Western blot results showed that compared with those in the NC group rats, the expression levels of GRP78 and ATF6 protein in the liver of the DM group rats were significantly increased, and the expression levels of GRP78 and ATF6 protein in the liver of the JPXZF intervention group rats were decreased, in a dosage-dependent manner. Compared with those in the DM + JL group rats, the expression levels of GRP78 and ATF6 protein in the liver of the DM + JH group rats were further decreased (*p* < 0.05) (Figures 2(b) and 2(c)).

The article "Mechanistic Research into the Effects of the Jianpi Xiaozhi Formula on Liver Injury in Diabetic Rats" was published in 2022. Journal: Evid Based Complement Alternat Med.

### 3.4. Effect of JPXZF on Autophagy

The results of RT-PCR showed that compared with that in the NC-group rats, the relative expression of Beclin-1 mRNA in the liver of the DM group rats was decreased significantly, while the relative expression of P62 mRNA was increased significantly. The relative expression of Beclin-1 mRNA in the liver of the JPXZF intervention group rats increased in a dosage-dependent manner compared with that in the DM group rats, and the relative expression of P62 mRNA was decreased, in a dosage-dependent manner, compared with that in the DM group. Compared with those in the DM + JL group rats, the relative expression levels of Beclin-1 mRNA in the liver of the DM + JH group rats was further increased, while the relative expression of P62 mRNA was further decreased (*p* < 0.05) (Figure 3(a)). The Western blot results showed that compared with those in the NC group rats, the expression levels of Beclin-1 and LC3II/I protein in the liver of the DM group rats were decreased significantly, while the expression level of P62 protein was increased significantly. The expression levels of Beclin-1 and LC3II/I protein in the liver of the JPXZF intervention group rats in increased in a dosage-dependent manner compared with those in the DM group rats, and the expression level of the P62 protein was decreased in a dosage-dependent manner. Compared with those in the DM + JL group rats, the expression levels of Beclin-1 protein in the liver of the DM + JH group rats were further increased, while the expression of P62 protein was decreased (*p* < 0.05) (Figures 3(b) and 3(c)).

The article "Mechanistic Research into the Effects of the Jianpi Xiaozhi Formula on Liver Injury in Diabetic Rats" was published in 2022. Journal: Evid Based Complement Alternat Med.

### 3.5. Effect of JPXZF on Autophagy Triggered by ERS

FAM134B expression is a biomarker of ER-autophagy. RT-PCR results showed that compared with that in the NC group rats, the relative expression of FAM134B mRNA in the liver of the DM group rats was decreased significantly, while the relative expression of FAM134B mRNA in the liver of the JPXZF intervention group rats was increased in a dosage-dependent manner. Compared with those in the DM + JL group rats, the relative expression levels of FAM134B mRNA in the liver of the DM + JH group rats were further increased (*p* < 0.05) (Figure 4(a)). The Western blot results showed that compared with that in the NC group rats, the expression level of FAM134B protein in the liver of the DM group rats was significantly lower, and the expression of FAM134B protein in the liver in the JPXZF intervention group of rats was increased in a dosage-dependent manner. Compared with those in the DM + JL group rats, the expression levels of FAM134B protein in the liver of the DM + JH group rats were further increased (*p* < 0.05) (Figures 4(b) and 4(c)). In addition, the immunofluorescence results were consistent with those of RT-PCR and WB (Figure 4(d)).

## 4. Discussion

The treatment of T2DM with NAFLD with either a Chinese medicine compound or a single drug has led to significant effects [32–34]. On the basis of many years of experience, Liuhuaizhen, the chief physician in our hospital who has proposed that JPXZF, which exerts the effects of both Jianpi Shugan and Huatan Quyu, is a valuable treatment for T2DM with NAFLD. Currently, the clinical treatment of T2DM with NAFLD mainly addresses symptoms and includes lifestyle changes and lipid-lowering intervention. However, after the liver function is impaired, lipid-lowering drugs are less effective. In this study, we observed that rat models of T2DM with NAFLD, which had been established by feeding a high-sugar and high-fat diet and STZ treatment, showed characteristics of hyperglycaemia, hyperlipidaemia, and hyperinsulinaemia. However, after JPXZF intervention, the rat levels of serum FBG, FINS, TG, and TC and rat body weight were obviously decreased. JPXZF was equally effective in treating T2DM with NAFLD; therefore, it is worthy of further study, including exploration into its mechanism of action.

NAFLD is one of the most common causes of chronic liver injury and abnormal liver enzyme levels. ALT and AST are the most commonly assessed biomarkers and representative enzymatic indexes for diagnosing liver diseases. ALT is mainly expressed in liver cell cytoplasm, and its enzymatic activity in liver is significantly higher than that in serum; therefore, a low rate of liver cell necrosis can lead to a significant increase in serum ALT levels. AST is mainly expressed in the mitochondria of liver cells. When large portions of liver tissues are necrotic, AST is released from mitochondria, and the serum AST level is significantly increased. However, the liver is an organ with strong preservation and regeneration ability. Small injuries to the liver are likely to be completely healed through the compensatory mechanisms in the liver, typically restoring liver function with no obvious dysfunction. In our research, the serum transaminase (ALT and AST) levels in the diabetic rats did not obviously increase, but the histopathological assays of the liver showed obvious pathological changes, including liver swelling, structural destruction, fatty degeneration, and inflammatory cell infiltration, which indicated that the liver of the diabetic rats had been injured. However, because the rats were in an early disease stage, only the histopathological changes were clear, with transaminase levels not yet increased; this pattern is consistent with the pathological evolution of NAFLD and can be the basis of study into early diabetic liver injury [35]. For many years, our research group has been devoted to clinical and animal experimental research into JPXZF treatments, and we have observed no adverse reactions, such as liver or kidney function damage or abnormal routine blood indexes [16, 19, 23]. In this study, after 8 weeks of intervention with JPXZF, no liver transaminase (ALT or AST) increased in the high-, intermediate-, and low-dosage groups. These results indicated that JPXZF induced no hepatotoxicity and was a safe and effective compound preparation in the rats.

The article "Mechanistic Research into the Effects of the Jianpi Xiaozhi Formula on Liver Injury in Diabetic Rats" was published in 2022. Journal: Evid Based Complement Alternat Med.

The pathology of T2DM in NAFLD is not clear, and ERS and autophagy are research hotspots. Under ERS, the ER protein GRP78 is released unfolded and chelated, activating PERK, IRE1*α*, and ATF6 [36]. Oxidative stress caused by foreign substances or the accumulation of unfolded or misfolded proteins in the ER can destroy ER homeostasis and lead to ERS, further aggravating the disorders in lipid metabolism and IR, exacerbating inflammatory reactions and increasing the cell apoptosis rate. Many factors interact to initiate lipid peroxidation, leading to excessive lipids deposition in the liver, which aggravates liver steatosis, damages the liver, and induces inflammatory lesions, indicating NAFLD. Zhu et al. [37] showed that ERS was involved in fatty degeneration induced by free fatty acids in the liver of rats with T2DM with NAFLD and that liraglutide might attenuate disordered lipid metabolism by suppressing the activation of ERS in liver tissue. Cheng et al. [38] established a transgenic MKR mouse model of T2DM with fatty liver by feeding the mice a high-fat diet and found that the TG and fatty acid levels in the liver of the model mice were significantly increased, and ERS markers GRP78, X-box binding protein 1 (XBP1), fatty acid synthase (FAS), acetyl-CoA carboxylase (ACC-*α*), and glycogen synthase kinase (GSK3*β*) mRNA expression levels were increased, which indicated that ERS was involved in regulating liver lipid metabolism and played an important role in the formation of fatty liver in T2DM. Our present study also revealed that a high-sugar and high-fat diet combined with STZ treatment induced the development of T2DM with NAFLD in rats and that these rats exhibited significantly increased relative mRNA and protein expression levels of GRP78 and ATF6, which indicated ERS in the model rats. With an increase in the dosage of the traditional Chinese medicine compound JPXZF, the relative mRNA and protein expression levels of GRP78 and ATF6 in the liver of the rats in each intervention group were decreased in a dosage-dependent manner, which indicated that JPXZF attenuated or prevented ERS in rats.

Autophagy involves the physiological degradation of material in mammals. ERS can induce autophagy, leading to the elimination of unnecessary proteins and restoring ER homeostasis [39]. Notably, ERS plays an important role in liver pathophysiology [40]. Recent evidence has shown that autophagy selectively degraded lipid droplets, and inhibiting autophagy increased the TG content in liver cells [41]. Therefore, autophagy and the accumulation of cellular lipids exert important impacts on the pathogenesis of NAFLD. He et al. [42] found that liraglutide, an analogue of glucagon-like peptide-1, induced autophagy and reduced the lipid accumulation in the livers of mice fed a high-fat diet. Electron microscopy revealed that after liraglutide treatment, the autophagy rate increased, the number of fat vacuoles decreased in the high-fat diet group, and p62 expression levels decreased significantly while those of LC3-II increased significantly. Zhang et al. [43] treated HepG2 liver cells with palmitic acid and found that the TG levels increased significantly; the protein expression of the ERS markers GRP78, p-PERK, ATF6, p-IRE1*α*, and XBP1s also increased significantly; the expression of the autophagy markers Beclin-1 and LC3-II/I decreased; the expression of p62 increased. After scutellarin intervention, the TG expression levels and the protein expression levels of the ERS markers GRP78, p-PERK, ATF6, p-IRE1*α*, and XBP1s all decreased significantly, and the expression levels of the autophagy markers Beclin-1 and LC3-II/I increased, and those of p62 decreased. Scutellarin thus attenuated liver lipid accumulation by promoting autophagy and reducing ERS. We also found that the expression levels of Beclin-1 and LC3II/I were decreased in T2DM with NAFLD model rats fed a high-sugar and high-fat diet and treated with STZ, but the expression levels of P62 were increased. After JPXZF treatment, the expression levels of Beclin-1 and LC3II/I increased, and the expression levels of P62 decreased, indicating that JPXZF promoted autophagy in the rats.

The article "Mechanistic Research into the Effects of the Jianpi Xiaozhi Formula on Liver Injury in Diabetic Rats" was published in 2022. Journal: Evid Based Complement Alternat Med.

ER-autophagy is one of the main pathways through which ER function is regulated because damaged ER, excess, insoluble or even toxic protein aggregates in cells are eliminated by autophagy, preventing disease. ER-autophagy may be involved in the pathogenesis and progression of IR, Parkinson's disease, and neuromuscular diseases [44–46]. Recent research has shown that FAM134B may be a receptor protein only in ER-autophagy because it does not localize to the healthy ER. Specifically, upon initiation of ER-autophagy, FAM134B was selectively located at the edge of the ER lamellar vesicle structure. Through its LC3-binding domain, FAM134B interacts with LC3/GABARAP to induce the fragmentation of ER lamellar vesicles and envelopment of the fragments by vesicles that deliver them to be degraded by hydrolases [47]. Xie et al. [48] found that the overexpression of FAM134B reduced ERS, reporting that the expression of C/-EBP homologous protein (CHOP) and GRP78 was decreased and that neuronal apoptosis was induced by epileptic seizures, but the downregulation of FAM134B expression led to the opposite effects. In addition, pretreatment with the selective autophagy inhibitor 3-methyladenine (3-MA) eliminated the effects of FAM134B on ERS and neuronal apoptosis. These results showed that FAM134B was an important regulator of ERS and neuronal apoptosis induced by epilepsy and exerted its effect by controlling autophagy. Li et al. [49] established a septic mouse model of myocardial injury by performing caecal ligation and puncture. Intervention with the autophagy inhibitor 3-MA significantly inhibited the expression of FAM134B and LC3-II/I and promoted myocardial ischaemic injury, inflammatory reactions, and cardiomyocyte apoptosis. Lipopolysaccharide (LPS) was used to induce cardiomyocytes. Overexpression of FAM134B significantly increased the expression of LC3-II/I and Beclin-1 and minimized the myocardial injury, inflammatory response, and apoptosis, while knocking out FAM134B expression led to the opposite effects. FAM134B-mediated ER-autophagy exerted a protective effect on septic myocardial injury in the mice by reducing inflammation and apoptosis. In our study, we found that a high-sugar and high-fat diet with STZ treatment-induced T2DM with NAFLD in rats, and through immunofluorescence assay, RT-PCR, and WB, we showed that the levels of FAM134B expression decreased in the model group and that the levels of FAM134B expression increased significantly after JPXZF treatment, which was consistent with the trend in the LC3II/I ratio change. All our experiments showed that JPXZF reduced ERS in rat models and that JPXZF enhanced ER-autophagy to reduce blood glucose and lipids levels, attenuate hyperinsulinaemia and reduce the number of fatty liver cells in T2DM with NAFLD rats.

The article "Mechanistic Research into the Effects of the Jianpi Xiaozhi Formula on Liver Injury in Diabetic Rats" was published in 2022. Journal: Evid Based Complement Alternat Med.

This study also had some limitations. First, JPXZF is a compound preparation comprising a variety of single traditional Chinese medicinal components, and the role each component plays in JPXZF treatment remains to be further studied. Second, short-term oral JPXZF administration does not result in liver function damage or other haemorheological changes, but the safety of long-term oral JPXZF use needs to be further assessed. Finally, JPXZF exerted its attenuating effects on T2DM with NAFLD by enhancing ER-autophagy; however, the mechanism through which FAM134B mediates ER-autophagy remains unknown, and further research is required.

## 5. Conclusions

In summary, ERS and autophagy are involved in the occurrence and development of T2DM with NAFLD and are important mechanisms in comorbidity pathogenesis. JPXZF enhances ER-autophagy, reduces blood glucose and lipid levels, attenuates hyperinsulinaemia, and reduces the degree of fatty deposits in hepatocytes by reducing ERS in T2DM with NAFLD models, providing new insights into the treatment of T2DM with NAFLD.

## Figures and Tables

**Figure 1:** Haematoxylin-eosin (HE) analysis of the rat liver: normal control (NC) group: healthy untreated rats; diabetes mellitus (DM) group: rat models of DM; DM + JL group: diabetic rats treated with low-dosage Jianpi Xiaozhi Formula (JPXZF) (4.5 g/kg/d); DM + JM group: diabetic rats treated with an intermediate JPXZF dosage (9 g/kg/d); DM + JH group: diabetic rats treated with high-dosage JPXZF (18 g/kg/d); DM + PBA group: diabetic rats treated with 4-phenylbutyric acid (PBA; 2.5 mg/kg/d).

**Figure 2:** Effects of Jianpi Xiaozhi Formula (JPXZF) on mRNA and protein expression associated with endoplasmic reticulum stress (ERS) in the rat models of type 2 diabetes mellitus (T2DM) with nonalcoholic fatty liver disease (NAFLD) induced by a high-sugar and high-fat diet combined with streptozotocin (STZ) treatment. Normal control (NC group): healthy untreated rats; diabetes mellitus (DM) group: rat models of DM; DM + JL group: diabetic rats treated with low-dosage Jianpi Xiaozhi formula (JPXZF) (4.5 g/kg/d); DM + JM group: diabetic rats treated with an intermediate dosage of JPXZF (9 g/kg/d); DM + JH group: diabetic rats treated with high-dosage JPXZF (18 g/kg/d); DM + PBA group: diabetic rats treated with 4-phenylbutyric acid (PBA; 2.5 mg/kg/d). (a) The mRNA expression levels of glucose-regulated protein 78/immunoglobulin-heavy-chain-binding protein (GRP78) and activating transcription factor 6 (ATF6) were assessed by quantitative real-time polymerase chain reaction; (b, c) GRP78 and ATF6 protein expression was determined by Western blotting (WB). The data are expressed as the means ± standard deviation. ^*∗*^*p* < 0.05 versus the NC group; ^#^*p* < 0 .05 versus the DM group; ^*c*^*p* < 0.05 versus the DM + JL group.

The article "Mechanistic Research into the Effects of the Jianpi Xiaozhi Formula on Liver Injury in Diabetic Rats" was published in 2022. Journal: Evid Based Complement Alternat Med.

**Figure 3:** Effects of Jianpi Xiaozhi Formula (JPXZF) on mRNA and protein expression associated with autophagy reaction in the rat model of type 2 diabetes mellitus (T2DM) with nonalcoholic fatty liver disease (NAFLD) induced by high sugar and high-fat diet combined with streptozotocin (STZ) treatment. Normal control (NC group): healthy untreated rats; diabetes mellitus (DM) group: rat models of DM; DM + JL group: diabetic rats treated with low-dosage Jianpi Xiaozhi formula (JPXZF) (4.5 g/kg/d); DM + JM group: diabetic rats treated with an intermediate dosage of JPXZF (9 g/kg/d); DM + JH group: diabetic rats treated with high-dosage JPXZF (18 g/kg/d); DM + PBA group: diabetic rats treated with 4-phenylbutyric acid (PBA; 2.5 mg/kg/d). (a) The mRNA expression levels of Beclin-1 and P62 were assessed by quantitative real-time polymerase chain reaction; (b, c) Beclin-1, P62, and long-chain 3II/I (LC3II/I) protein expressions were determined by Western blotting (WB). The data are expressed as the means ± standard deviation.^*∗*^*p* < 0.05 versus NC group; ^#^*p* < 0 .05 versus DM group; ^*c*^*p* < 0.05 versus DM + JL group.

**Figure 4:** Effects of Jianpi Xiaozhi formula (JPXZF) on mRNA and protein expression associated with endoplasmic reticulum stress (ERS)-autophagy in rat models of type 2 diabetes mellitus (T2DM) with nonalcoholic fatty liver disease (NAFLD) induced by a high-sugar and high-fat diet combined with streptozotocin (STZ) treatment. Normal control (NC group): healthy untreated rats; diabetes mellitus (DM) group: rat models of DM; DM + JL group: diabetic rats treated with low-dosage Jianpi Xiaozhi formula (JPXZF) (4.5 g/kg/d); DM + JM group: diabetic rats treated with an intermediate dosage of JPXZF (9 g/kg/d); DM + JH group: diabetic rats treated with high-dosage JPXZF (18 g/kg/d); DM + PBA group: diabetic rats treated with 4-phenylbutyric acid (PBA; 2.5 mg/kg/d). (a) The mRNA expression levels of family with sequence similarity 134, member B (FAM134B) were assessed by quantitative real-time polymerase chain reaction. (b, c) FAM134B protein expression was determined by Western blotting (WB). (d) Immunofluorescence image analysis showed the relative expression levels of FAM134B in the rat liver. The nucleus showed blue fluorescence emitted by DAPI. The target protein FAM134B was labelled with green fluorescence. The data are expressed as the means ± standard deviation. ^*∗*^*p* < 0.05 versus the NC group; ^#^*p* < 0 .05 versus the DM group; ^*c*^*p* < 0.05 versus the DM + JL group.

The article "Mechanistic Research into the Effects of the Jianpi Xiaozhi Formula on Liver Injury in Diabetic Rats" was published in 2022. Journal: Evid Based Complement Alternat Med.

**Table 1:** Comparison of general serological indexes of the rats in different groups after 8 weeks of JPXZF intervention.

Groups	NC group	DM group	DM + JL group	DM + JM group	DM + JH group	DM + PBA group
FBG (mmol/L)	4.83 ± 0.19	11.57 ± 0.68^a^	11.33 ± 0.58^a^	11.19 ± 0.50^a^	5.43 ± 0.60^abc^	5.38 ± 0.49^abc^
FINS (uIU/mL)	18.89 ± 2.21	30.02 ± 6.82^a^	24.75 ± 5.53^ab^	22.72 ± 4.01^b^	19.82 ± 2.48^bc^	22.98 ± 4.09^b^
TG (mmol/L)	0.90 ± 0.10	3.09 ± 0.24^a^	2.90 ± 0.16^ab^	1.99 ± 0.96^ab^	1.50 ± 0.17^abc^	1.97 ± 0.10^abc^
TC (mmol/L)	3.57 ± 0.38	6.54 ± 0.34^a^	6.44 ± 0.29^a^	6.25 ± 0.24^a^	5.71 ± 0.30^abc^	6.03 ± 0.17^abc^
ALT (U/L)	40.64 ± 4.24	44.32 ± 7.69	44.54 ± 7.77	42.67 ± 6.22	43.28 ± 6.77	42.03 ± 5.76
AST (U/L)	46.17 ± 3.25	48.29 ± 3.96	49.10 ± 5.00	46.70 ± 4.66	47.59 ± 3.79	48.82 ± 2.35
Body weight (g)	345.5 ± 10.39	428.13 ± 40.20^a^	394.38 ± 35.73^ab^	373.88 ± 31.90^b^	352.88 ± 18.26^bc^	374.25 ± 30.16^b^

Normal control (NC) group: healthy untreated rats; diabetes mellitus (DM) group: rat models of DM; DM + JL group: diabetic rats treated with low-dosage Jianpi Xiaozhi Formula (JPXZF) (4.5 g/kg/d); DM + JM group: diabetic rats treated with an intermediate JPXZF dosage (9 g/kg/d); DM + JH group: diabetic rats treated with high-dosage JPXZF (18 g/kg/d); and DM + PBA group: diabetic rats treated with 4-phenylbutyric acid (PBA; 2.5 mg/kg/d). FBG, fasting blood glucose; FINS, fasting insulin; TG, triglyceride; TC, total cholesterol; ALT, alanine aminotransferase; AST, aspartic acid aminotransferase. The data are expressed as the means ± standard deviation. ^*a*^*p* < 0.05 compared with the NC group; ^*b*^*p* < 0.05 compared with the DM group; ^*c*^*p* < 0.05 compared with the DM + JL group.

## Data Availability

All the data generated or analysed during this study are included in the article. The data that support this study are available from the corresponding author only upon reasonable request after the study has been published.

The article "Mechanistic Research into the Effects of the Jianpi Xiaozhi Formula on Liver Injury in Diabetic Rats" was published in 2022. Journal: Evid Based Complement Alternat Med.

## Abbreviations

NAFLD: Nonalcoholic fatty liver disease
T2DM: Type 2 diabetes mellitus
DM: Diabetes mellitus
NASH: Nonalcoholic steatohepatitis
IR: Insulin resistance
JPXZF: Jianpi Xiaozhi formula
RT-PCR: Reverse-transcription polymerase chain reaction
WB: Western blotting
HE: Haematoxylin-eosin
STZ: Streptozotocin
ERS: Endoplasmic reticulum stress
ER: Endoplasmic reticulum
FBG: Fasting blood glucose
TG: Triglyceride
TC: Total cholesterol
ALT: Alanine aminotransferase
AST: Aspartic acid aminotransferase
FINS: Fasting insulin
GRP78: Glucose-regulated protein 78
ATF6: Activating transcription factor 6
FAM134B: Family with sequence similarity 134 member B
LC3II/I: Light chain 3II/I
SD: Standard deviation.
